The article "Biodegradation of the Allelopathic Chemical m-Tyrosine by Bacillus aquimaris SSC5 Involves the Homogentisate Central Pathway" was retracted in 2014. Reasons: fabricated or falsified data; fabricated or falsified results; concerns about the data.

# Biodegradation of the Allelopathic Chemical *m*-Tyrosine by *Bacillus aquimaris* SSC5 Involves the Homogentisate Central Pathway

**DOI:** 10.1371/journal.pone.0075928

**Published:** 2013-10-01

**Authors:** Fazlurrahman Khan, Munesh Kumari, Swaranjit Singh Cameotra

**Affiliations:** Institute of Microbial Technology, Council of Scientific and Industrial Research (CSIR), Chandigarh, India; University Medical Center Utrecht, The Netherlands

## Abstract

*m*-Tyrosine is an amino acid analogue, exuded from the roots of fescue grasses, which acts as a potent allelopathic and a broad spectrum herbicidal chemical. Although the production and toxic effects of *m*-tyrosine are known, its microbial degradation has not been documented yet. A soil microcosm study showed efficient degradation of *m*-tyrosine by the inhabitant microorganisms. A bacterial strain designated SSC5, that was able to utilize *m*-tyrosine as the sole source of carbon, nitrogen, and energy, was isolated from the soil microcosm and was characterized as *Bacillus aquimaris*. Analytical methods such as HPLC, GC-MS, and ^1^H-NMR performed on the resting cell samples identified the formation of 3-hydroxyphenylpyruvate (3-OH-PPA), 3-hydroxyphenylacetate (3-OH-PhAc), and homogentisate (HMG) as major intermediates in the *m*-tyrosine degradation pathway. Enzymatic assays carried out on cell-free lysates of *m*-tyrosine-induced cells confirmed transamination reaction as the first step of *m*-tyrosine degradation. The intermediate 3-OH-PhAc thus obtained was further funneled into the HMG central pathway as revealed by a hydroxylase enzyme assay. Subsequent degradation of HMG occurred by ring cleavage catalyzed by the enzyme homogentisate 1, 2-dioxygenase. This study has significant implications in terms of understanding the environmental fate of *m*-tyrosine as well as regulation of its phytotoxic effect by soil microorganisms.

## Introduction

*m*-Tyrosine is a non-proteinogenic amino acid analogue with phytotoxic properties that is exuded from the roots of fine fescue grasses to grant a competitive advantage over other plants [1], [2], [3], [4]. *m*-Tyrosine also arises from the oxidation of L-phenylalanine by hydroxyl radicals and peroxynitrite [5], [6]. The phytotoxic activity of *m*-tyrosine is due to its inhibitory effects on the root development of competing plants [1]. Similarly, *m*-tyrosine also inhibits growth of prokaryotic cells, *Escherichia coli* and *Bacillus* sp. [7], [8], [9]. Previous studies showed that the cytotoxic effects of *m*-tyrosine is the result of its misincorporation into cellular protein in place of phenylalanine [10], [11], [12], [13]. The accumulation of *m*-tyrosine in mammalian tissues is used as an indicator for determining the oxidative stress and aging process [14], [15]. Several bacteria, e. g. *Streptomyces* spp., use *m*-tyrosine as a precursor for the synthesis of antibiotics such as mureidomycins, pacidamycins, and napsamycins [16]. Plant roots exude various allelochemicals to compete with other plants; however, soil microorganisms residing nearby the roots influence their phytotoxic effects either by co-metabolic transformation or utilizing them as sole carbon, nitrogen, and energy sources [17], [18], [19]. Thus, soil microorganisms can either enhance or decrease the phytotoxic properties of allelochemicals which interferes with defense properties of *m*-tyrosine producing plants. In some cases, the microbial degradation products of the allelopathic chemicals pose potential phytotoxic effects, while some of the microbially transformed products of allelochemicals decrease their level of phytotoxic effect as compared to the original compounds [3], [18], [19], [20], [21], [22], [23], [24], [25]. Several studies reported microbial degradation of previously characterized allelochemicals such as sorgoleone, juglone, benzoxazinoids, and other flavonoids [26], [27], [28], [29], while there is no information available on the degradation of *m*-tyrosine by means of bacterial isolates.

The article "Biodegradation of the Allelopathic Chemical m-Tyrosine by Bacillus aquimaris SSC5 Involves the Homogentisate Central Pathway" was retracted in 2014. Reasons: fabricated or falsified data; fabricated or falsified results; concerns about the data.

The present study shows the isolation and characterization of an aerobic bacterium from a soil microcosms set up for the degradation of *m*-tyrosine. The strain *Bacillus aquimaris* SSC5 isolated from a soil microcosm utilizes *m*-tyrosine as the sole source of carbon, nitrogen, and energy. The resting cell studies and enzyme assays confirm the formation of 3-OH-PPA, 3-OH-PhAc, and HMG as the major metabolic intermediates. Based on the above studies we conclude that the degradation of *m*-tyrosine occurs via the homogentisate central pathway in *Bacillus aquimaris* SSC5.

## Materials and Methods

### Chemicals and growth media

Analytical grade *m*-tyrosine (>98% purity), 3-hydroxyphenylacetic acid (>99% purity), and homogentisate (98% purity) were purchased from Sigma-Aldrich (St, Louis, MO, USA). Minimal salt medium (MSM) used in the present study was prepared as described earlier [30], with a minor modification i.e. absence of nitrogen source [(NH_4_)_2_SO_4_]. Nutrient agar (NA) and nutrient broth (NB) both at one-quarter strength (1/4^th^) were used for bacterial growth and culture maintenance.

### *m*-Tyrosine degradation in soil microcosms

The rhizosphere soil samples of fine fescue grasses (*Festuca rubra* ssp. *commutata*) were collected from the lawn of the Institute of Microbial Technology, Chandigarh, India. The soil pH, moisture, total organic carbon, and total nitrogen were 6.4, 5.2%, 3.2%, and 4.7%, respectively. Before their use in inoculating the microcosms, the soil samples were sieved through a 2 mm mesh for the removal of stones and debris. Soil microcosms studies were carried out as described previously with minor modifications [31]. Subsequently, 10 g soil sample was suspended in 50 ml MSM in a 250-ml Erlenmeyer flask supplemented with 200 µM *m*-tyrosine. The above microcosms were also supplemented with or without (i) 10 mM glucose and 5 mM succinate as the sole carbon source, or (ii) 0.8 g l^−1^ NH_4_Cl as the sole nitrogen source, or (iii) 10 mM glucose, 5 mM succinate and 0.8 g l^−1^ NH_4_Cl as the sole carbon and nitrogen source. A control was also set up containing 10 g autoclaved soil in 50 ml MSM and *m*-tyrosine (200 µM). Further, these flasks were incubated at 30°C under shaking condition at 150 rpm. Samples were withdrawn from the test and control flasks at regular intervals and analyzed for the disappearance of *m*-tyrosine. All experiments were carried out in triplicate.

The article "Biodegradation of the Allelopathic Chemical m-Tyrosine by Bacillus aquimaris SSC5 Involves the Homogentisate Central Pathway" was retracted in 2014. Reasons: fabricated or falsified data; fabricated or falsified results; concerns about the data.

### Isolation and identification of *m*-tyrosine degrading bacteria

The soil slurries that mediated complete degradation of *m*-tyrosine were serially diluted and spread plated on 1/4^th^-diluted nutrient agar (1/4-NA) and a selective media (MSM-agar supplemented with 500 µM *m*-tyrosine). Following seven days of incubation, the bacterial colonies that appeared on the agar were selected for characterization and were tested for *m*-tyrosine degradation. Initial screening was performed by inoculating selected bacterial colonies in 10 ml McCartney vials containing 5 ml carbon-free MSM supplemented with different concentrations (50–500 µM) of *m*-tyrosine. Bacterial growth, along with the measurement of the amount of ammonia released and depletion of substrate were used as an indicator for positive degrading activity as described earlier for 4-nitroaniline and 2-chloro-4-nitroaniline degradation studies [32], [33]. Further, the efficient *m*-tyrosine degrading strain was identified using polyphasic taxonomy and 16S rRNA gene sequencing as described earlier [34]. The 16S rRNA gene sequence (1375 bp) of strain SSC5 was compared to those of the type strains of *Bacillus* using the BLAST search function of EzTaxon server version 2.1 (www.eztaxon.org).

### Growth studies and degradation of *m*-tyrosine by strain SSC5

The growth studies of strain SSC5 were performed in 50 ml carbon-free MSM supplemented with different concentrations (50–500 µM) of *m*-tyrosine by inoculating (1%, v/v) overnight seed culture grown in 1/4-NB. Cultures were incubated on a rotary shaker at 200 rpm at 30°C. After every 8 hours, cultures were withdrawn and optical cell density was monitored at 600 nm using Lambda EZ 201 UV-visible spectrophotometer (Perkin-Elmer Inc, USA). Bacterial growth was also monitored by measuring the total protein of the cultures with the Pierce BCA protein assay kit (Thermo Scientific, USA) according to the procedure as described earlier [32], [33]. The culture fluid samples were centrifuged at 8,000× g for 10 min to obtain cell-free supernatants which were used for the analysis of the amount of ammonia released, depletion of *m*-tyrosine, and identification of intermediates using the method described later. An un-inoculated flask and a flask that was inoculated with heat-killed cells of strain SSC5 were used as abiotic and negative controls respectively. Another control experiment was also conducted by inoculating strain SSC5 in carbon-free MSM only.

The article "Biodegradation of the Allelopathic Chemical m-Tyrosine by Bacillus aquimaris SSC5 Involves the Homogentisate Central Pathway" was retracted in 2014. Reasons: fabricated or falsified data; fabricated or falsified results; concerns about the data.

### Resting cell studies

In order to identify the metabolic intermediates of *m*-tyrosine catabolic pathway in strain SSC5, a resting cell study was carried out according to the method described elsewhere [35]. A volume of 1.6 liter of 1/4-NB supplemented with *m*-tyrosine (300 µM) was inoculated with an overnight 1/4-NB grown seed culture (6%, v/v) of strain SSC5 and was incubated at 30°C under shaking at 200 rpm up to 24 hours. When the optical density (OD_600_) of the culture reached 1.3–1.4, the induced cells were harvested by centrifugation at 8,000× g at room temperature for 10 min, washed twice with sodium phosphate buffer (20 mM, pH 7.2) and suspended in 100 ml of carbon-free MSM. This suspension was divided into four aliquots of 25 ml each. First two aliquots with heat killed cells (by incubating in boiling water for 30 min) and without heat killed cells not supplemented with *m*-tyrosine were used as negative controls, respectively. The heat killed cells supplemented with *m*-tyrosine in third aliquot was used as another control. The fourth aliquot supplemented with 300 µM *m*-tyrosine was used as test. Similarly, the resting cell studies on 3-OH-PhAc and HMG were also carried out with the *m*-tyrosine grown cells of strain SSC5. Each flask was incubated at 30°C with shaking at 200 rpm. Samples (2.0 ml) were withdrawn from both control and experimental flasks at regular intervals of 2 hours and were analyzed for the amount of ammonia released, followed by High Performance Liquid Chromatography (HPLC), Gas-Chromatography Mass-Spectroscopy (GC-MS) and ^1^H-nuclear magnetic resonance (^1^H-NMR) spectra analysis (methods described later).

### Enzyme assays with cell-free lysates

*m*-Tyrosine-induced cells of strain SSC5 were harvested by centrifugation, washed twice and suspended in the sodium phosphate buffer (20 mM, pH 7.2). The cell suspensions lysed by passages through a French pressure cell (20,000 lb/in^2^) were centrifuged at 12,000 rpm for 30 min at 4°C and supernatant was separated to obtain cell-free extract. The cell-free ectract was used for determing activities of transaminase, hydroxylase, and homogentisate 1, 2-dioxygenase, respectively as described below. Protein content of the cell-free extracts was determined with the Pierce BCA protein assay kit (Thermo Scientific, USA).

The article "Biodegradation of the Allelopathic Chemical m-Tyrosine by Bacillus aquimaris SSC5 Involves the Homogentisate Central Pathway" was retracted in 2014. Reasons: fabricated or falsified data; fabricated or falsified results; concerns about the data.

### Transaminase enzyme assay

The enzyme assay, for the transamination reaction from the cell-free lysates of strain SSC5, was carried out according to the method described earlier with minor modifications [36], [37]. One ml reaction volume contained sodium phosphate buffer (20 mM, pH 7.0), 100 µM α-ketoglutarate (α-KG), 25 µM pyridoxal phosphate, cell-free lysate (0.5 mg ml^−1^ of total protein), and 100 µM *m*-tyrosine. Transamination reaction was also carried out by taking the cell-free lysates prepared from the glucose grown cells. The transamination reactions were initiated by adding 100 µM *m*-tyrosine to the reaction mixture and incubated at 30°C. Enzyme activity was calculated based on substrate depletion as determined by HPLC. The reactions that lacked either α-KG or cell-free lysates prepared from cells of strain SSC5 grown with *m*-tyrosine or glucose were used as controls.

### Hydroxylase enzyme assay

It has been reported that the formation of homogentisate (HMG) from 3-hydroxyphenylacetate (3-OH-PhAc) occurs by the action of 3-hydroxyphenylacetate 6-hydroxylase [38], [39]. The hydroxylase assay was carried out as described previously with minor modifications [40]. One ml reaction volume contained sodium phosphate buffer (20 mM, pH 7.0), 100 µM 3-OH-PhAc, 200 µM NADH, 50 µM FAD, and cell-free lysate (0.5 mg ml^−1^ of total protein). The hydroxylase reaction was initiated by adding 100 µM 3-OH-PhAc to the reaction mixture and incubated at 25°C. The control reactions lacking either substrate or cell-free lysate were also used during the above reaction. Substrate depletion and product formation was quantified by HPLC. The enzyme specific activity was determined based on the substrate depletion in the reaction mixture.

### Homogentisate 1, 2-dioxygenase enzyme assay

The homogentisate 1, 2-dioxygenase activity in the cell-free lysate was determined spectrophotometrically by measuring the formation of maleylacetoacetate (MA) at 330 nm as described previously [41], [42]. The specific activity was calculated with the help of molar extinction coefficient of MA, 13,500/M/cm [43]. One ml reaction volume contained sodium phosphate buffer (20 mM, pH 7.0), 50 µM FeSO_4_, 2 mM ascorbate, cell-free lysate (0.5 mg ml^−1^ of total protein), and 100 µM HMG. Similarly, another reaction was carried out with addition of cell-free lysate prepared either from the glucose or 3-OH-PhAc grown cells. The reactions were initiated by adding 100 µM HMG to the mixture and incubated at 30°C. The enzyme activity was determined spectrophotometrically by measuring the absorbance at a wavelength of 330 nm at a time interval of 1 min using Lambda EZ 201 UV-visible spectrophotometer (Perkin-Elmer Inc, Massachusetts, USA). Reactions without cell-free lysate was set up as negative control.

The article "Biodegradation of the Allelopathic Chemical m-Tyrosine by Bacillus aquimaris SSC5 Involves the Homogentisate Central Pathway" was retracted in 2014. Reasons: fabricated or falsified data; fabricated or falsified results; concerns about the data.

### Analytical methods

Ammonia concentration was monitored by a colorimetric method using the ‘Ammonia Estimation Kit’ (Sigma Aldrich, USA) according to the manufacturers' recommendations. The brown color pigment formation in the media was quantified by measuring the optical density at 400 nm in spectrophotometer as previously reported [44]. Similarly, the quantitative measurement of *m*-tyrosine degradation and identification of metabolic intermediates were analyzed by HPLC as per the method described earlier with minor modifications [3]. Samples (2.0 ml) from soil microcosms were withdrawn at regular time intervals and centrifuged for 10 min at 5,000 rpm. The clear supernatants were filtered with 0.2 µm membrane filters (Millipore Inc. USA) and analyzed by HPLC. Similarly, the cell-free aqueous culture supernatants collected from growth studies, resting cell studies, and enzyme assays were also filtered and analyzed by HPLC. The HPLC used for the sample analysis was a Waters HPLC system (Waters, USA) equipped with a UV detector and a RP-C18/Lichrospher 5-µM column. The mobile phase and the flow rate were the same as described by Kaur et al. [3]. The peaks of eluents were monitored at 280 nm. *m*-Tyrosine as well as its metabolic intermediates were quantified using calibration curves made with authentic standards. Further, the identified and unidentified metabolic intermediates detected from the samples of resting cell studies were also analyzed by GC-MS and ^1^H-NMR. For the GC-MS analysis, samples were prepared by mixing an equal volume of ethyl acetate to the cell-free aqueous culture and liquid-liquid extraction was performed by layer separation sequentially at neutral and acidic pH. The extracted organic phase was pooled and dried under nitrogen flow using RotaVapor II (BUCHI, Switzerland). The derivatization of metabolic intermediates in the sample was performed by using bis(trimethylsilyl)-trifluoroacetamide as previously described [45]. The derivatized samples were analyzed by GC-MS using QP2010S (Shimadzu Scientific Instruments, USA) with temperature program and other parameters used for GC analysis as reported previously [46]. ^1^H-NMR spectra of putatative intermediates were recorded using Bruker Avance DRX-300 spectrometer (Bruker, Germany) according to the method described earlier [47]. The dried extracted sample was dissolved in deuterated chloroform (CDCl_3_) in 5-mm NMR tubes and the spectra was recorded at 300 MHz. The chemical shift (δ) is given in parts per million (ppm) relative to tetramethylsilane (TMS) as internal standard.

The article "Biodegradation of the Allelopathic Chemical m-Tyrosine by Bacillus aquimaris SSC5 Involves the Homogentisate Central Pathway" was retracted in 2014. Reasons: fabricated or falsified data; fabricated or falsified results; concerns about the data.

### Nucleotide sequence

A total of 1375 base pairs of the 16S rRNA gene of strain SSC5 were sequenced. This sequence has been deposited to GenBank with accession no. KC607748.

## Results

### Degradation of *m*-tyrosine in soil microcosms

Samples collected from the soil microcosms were analyzed by HPLC in order to determine the degradation kinetics of *m*-tyrosine. Degradation of *m*-tyrosine in carbon-amended soil microcosms was initiated with a lag phase of ∼2 days, and thereafter the rate of degradation increased and was completed within 6 days of incubation (Figure 1). In contrast, degradation of *m*-tyrosine in the unamended soil microcosms was slower (Figure 1). The rate of *m*-tyrosine degradation was much slower in microcosms amended with only nitrogen (NH_4_Cl) or with a combination of nitrogen and carbon when compared to the above carbon-amended or unamended set ups (Figure 1). This difference in the rate of *m*-tyrosine degradation in soil microcosms was likely because the microorganisms utilized more the more favorable nitrogen source NH_4_Cl. No transformation of *m*-tyrosine was observed in the sterile soil (Figure 1). The above results clearly indicate that the soil microorganims utilized *m*-tyrosine as sole source of carbon, nitrogen, and energy

**Figure 1:** Biotransformation of *m*-tyrosine in soil microcosms under aerobic conditions. (▪), carbon-amended; (○), unamended; (Δ), nitrogen-amended; (•), carbon and nitrogen-amended; (□), sterile. Values are presented as arithmetic mean of data obtained from experiments carried out in triplicate; error bars represent standard deviation.

### Isolation and characterization of *m*-tyrosine degrading bacteria

Fifteen morphologically different colonies were isolated from the soil microcosms. These isolates were further screened for their ability to utilize *m*-tyrosine as the sole source of carbon, nitrogen, and energy . Among these isolates, one strain designated SSC5 was found to be an efficient *m*-tyrosine degrader and therefore was further studied to characterize its *m*-tyrosine degradation pathway.

Strain SSC5 was found to be Gram variable, endospore forming, aerobic, catalase positive, and oxidase negative. The colonies were pale orange-yellow in color, slightly raised with irregular edges observed after overnight incubation on NA at 30°C. The optimal growth temperature and pH were 30–37°C and 6.0–7.0, respectively. This strain produced acid from D-fructose, D-glucose, maltose, D-ribose, sucrose, and D-trehalose. The strain efficiently hydrolyzed casein, starch and Tween 80; however, it was not capable of hydrolyzing aesculin, hypoxanthine, xanthine, and tyrosine. The above data identifies strain SSC5 as closely related to *Bacillus aquimaris* TF-12 [48]. Strain SSC5 utilized acetate, glucose, and succinate as sole carbon sources. The partial 16S rRNA gene sequence (1375 bp) of strain SSC5 showed 99% sequence similarity to that of *Bacillus aquimaris* strain TF-12. Thus, based on the morphological and physiological characteristics and phylogenetic analysis, strain SSC5 was identified as *Bacillus aquimaris* SSC5.

The article "Biodegradation of the Allelopathic Chemical m-Tyrosine by Bacillus aquimaris SSC5 Involves the Homogentisate Central Pathway" was retracted in 2014. Reasons: fabricated or falsified data; fabricated or falsified results; concerns about the data.

### Growth and degradation of *m*-tyrosine by strain SSC5

A growth study of strain SSC5 was carried out using different concentrations of *m*-tyrosine ranging from 50 to 500 µM. Growth of strain SSC5 was completely abolished at an *m*-tyrosine concentration of 400 µM , whereas 300 µM of *m*-tyrosine was found to be optimal for its growth. Strain SSC5 experienced a lag phase of ∼10 hours during its growth in carbon-free MSM supplemented with 300 µM *m*-tyrosine (Figure 2). Following lag phase, SSC5 grew exponentially, as determined by the increase of total cell protein up to the value of 9.6 µg ml^−1^. The increase in growth was accompanied by a decrease in the concentration of *m*-tyrosine. The complete depletion of *m*-tyrosine was observed at 48 hours of incubation (Figure 2). Although, no metabolic intermediates were identified during the growth study, a slight accumulation of ammonia (84 µM) was observed (Figure 2). This non-stoichiometric release of ammonia suggested that *m*-tyrosine might possibly be utilized as the sole nitrogen source for the growth of strain SSC5. The above results are in close agreement with the results reported earlier on the degradation of 3-nitrotyrosine by *Burkholderia* sp. strain JS165 and *Variovorax paradoxus* JS171 [36]. Growth yield of strain SSC5 on *m*-tyrosine was found to be 0.35 g of cells/g of *m*-tyrosine. The rate of *m*-tyrosine degradation by strain SSC5 during the growth studies was calculated to be 8.6 nmol min^−1^ mg of protein^−1^. Strain SSC5 was unable to grow in MSM in the absence of *m*-tyrosine as well as in MSM supplemented with L-tyrosine. Thus, the above results indicated that *m*-tyrosine is being utilized as the sole source of carbon, nitrogen, and energy by strain SSC5.

The article "Biodegradation of the Allelopathic Chemical m-Tyrosine by Bacillus aquimaris SSC5 Involves the Homogentisate Central Pathway" was retracted in 2014. Reasons: fabricated or falsified data; fabricated or falsified results; concerns about the data.

**Figure 2:** Growth of *Bacillus aquimaris* SSC5 on *m*-tyrosine as the sole carbon, nitrogen, and energy source. (•), *m*-tyrosine; (▴), total protein; (○), NH_4_^+^. Values are presented as arithmetic mean of data obtained from experiments carried out in triplicate; error bars represent standard deviation.

### Elucidation of catabolic pathway for *m*-tyrosine degradation by strain SSC5

During the growth study, no putative metabolic intermediates of *m*-tyrosine degradation were identified; therefore, samples from resting cell studies and enzyme assays were analyzed for the identification of intermediates. Previous studies on the bacterial degradation of L-tyrosine have shown that the first step of degradation is the transamination reaction which results in the formation of 4-hydroxyphenylpyruvate (4-OH-PPA), which subsequently undergoes degradation either by the homogentisate (HMG) or the homoprotocatechuate (HPC) central pathway [38], [49]. HPLC analysis of the samples from the resting cell study using *m*-tyrosine induced cells showed the presence of three additional compounds, eluting at 4.82, 6.36, and 8.10 min, respectively (Figure 3A). Peaks with the retention time (R*t*) of 6.36 and 8.10 min, corresponded to the authentic standards of 3-hydroxyphenylacetate (3-OH-PhAc) and HMG, respectively. However, the peak with an R*t* value of 4.82 min was not identified. In the subsequent GC-MS analysis, these compounds were eluted at 10.94 (3-OH-PhAc), 12.22 (unknown intermediate), and 15.85 min (HMG), respectively (Figure 3B). The unknown intermediate (R*t*, 12.22 min; m/z 324) was identified as 3-hydroxyphenylpyruvate (3-OH-PPA) on the basis of mass fragmentation pattern in GC-MS analysis (Figure 4). The identities of 3-OH-PhAc (R*t*, 10.94 min; m/z 296) and HMG (R*t*, 15.85 min; m/z 384) intermediates were also confirmed by mass fragmentation pattern analysis (Figure 4). The formation of 3-OH-PPA as a *m*-tyrosine degradation pathway intermediate was confirmed by ^1^H-NMR analysis. The ^1^H-NMR analysis showed appearance of two broadened singlets of hydroxyl proton, one from carboxylic acid (COOH) and another from aromatic hydroxyl (C-3-OH) with the chemical shift values of 5.0 and 11.0 ppm, respectively (Figure 5). Similarly, two singlets appeared with the chemical shift values of 4.78 and 6.53 ppm showing the presence of methylene proton (CH_2_) and benzene proton (C-2-H) (Figure 5). Three doublet of doublets appeared at 6.54, 6.62, and 6.97 ppm which corresponded with the chemical shift values of benzene protons at position C-4, C-5, and C-6, respectively (Figure 5). The above ^1^H-NMR results confirmed the formation of 3-OH-PPA as the first metabolic intermediate of *m*-tyrosine degradation.

The article "Biodegradation of the Allelopathic Chemical m-Tyrosine by Bacillus aquimaris SSC5 Involves the Homogentisate Central Pathway" was retracted in 2014. Reasons: fabricated or falsified data; fabricated or falsified results; concerns about the data.

**Figure 3:** Representative HPLC and GC-MS chromatograms of intermediates identified during the degradation of *m*-tyrosine by resting cells of *Bacillus aquimaris* SSC5. (A) HPLC chromatograms of intermediates identified at different time intervals. (B) GC-MS chromatograms of TMS-derivatized authentic standards and the identified intermediates. Peaks at R*t* values correspond to: 5.62 min = *m*-tyrosine with m/z 325; 10.94 min = 3-OH-PhAc with m/z 296; 12.22 min = 3-OH-PPA with m/z 324; 15.85 min = HMG with m/z 384.

**Figure 4:** Mass fragmentation patterns of *m*-tyrosine intermediates including 3-OH-PPA, 3-OH-PhAc, and HMG analyzed by GC-MS.

**Figure 5:** ^1^H-NMR analysis of the 3-hydroxyphenylpyruvate (3-OH-PPA) intermediate indentified during the degradation of *m*-tyrosine by resting cells of *Bacillus aquimaris* SSC5.

*m*-Tyrosine-induced cells of strain SSC5 completely degraded *m*-tyrosine within 8 hours of incubation with the appearance and disappearance of intermediates namely 3-OH-PPA, 3-OH-PhAc, and HMG (Figure 6A). Thus, results from the resting cell study established that the degradation of *m*-tyrosine occurs with the formation of 3-OH-PPA and 3-OH-PhAc as intermediates, which are subsequently transformed into HMG. The induced cells of strain SSC5 also degraded 3-OH-PhAc via the formation of HMG as an intermediate and the complete degradation of 3-OH-PhAc occurred after 12 hours of incubation (Figure 6B). Similarly, HMG was degraded completely by the same cells after 8 hours of incubation (Figure 6C). Boiled cells were used as a control for the experiment related to HMG degradation and a brown color was observed in the medium, whereas there was no such color formation in the test samples (Figure 6C). The above results suggested that the dead (heat-inactivated) cells could not transform HMG, leading to the accumulation of HMG in the culture medium. Upon chemical oxidation and polymerization of HMG, pyomelanin pigments were formed that turned the color of the medium brown [44], [50]. This phenomenon has been described previously by Mendez et al. [42]. Previous reports also showed that the mutational inactivation of pathway gene(s) responsible for the catabolism of HMG, results in the formation of brown pigments due to accumulation of HMG and its chemical oxidation [38], [51], [52]. Our results provide evidence that the degradation of *m*-tyrosine occurs via the central pathway of HMG degradation.

**Figure 6:** Degradation kinetics of *m*-tyrosine, 3-hydroxyphenylacetate, and homogentisate by *m*-tyrosine-induced cells of strain SSC5. (A) *m*-Tyrosine degradation kinetics. (•), *m*-tyrosine; (○), 3-OH-PPA; (Δ), 3-OH-PhAc; (▴), HMG; (▪), *m*-tyrosine in abiotic control. (B) 3-Hydroxyphenylacetate degradation kinetics. (•), 3-OH-PhAc; (▪), HMG. (C) Homogentisate degradation kinetics. (•), HMG; (○), brown color (as measured by the OD_400_) in control. Values are presented as arithmetic mean of data obtained from experiments carried out in triplicate; error bars represent standard deviation.

The article "Biodegradation of the Allelopathic Chemical m-Tyrosine by Bacillus aquimaris SSC5 Involves the Homogentisate Central Pathway" was retracted in 2014. Reasons: fabricated or falsified data; fabricated or falsified results; concerns about the data.

### *m*-Tyrosine transaminase activity

Previous studies have shown that the first step of L-tyrosine degradation occurs by transamination reaction with the formation of 4-OH-PPA [38]. Thus, the identification of the 3-OH-PPA intermediate during the resting cell study leads us to posit that the first step of *m*-tyrosine degradation is also initiated with a transamination reaction. The transaminase enzyme assay from the cell-free lysates prepared from the *m*-tyrosine grown cells showed the accumulation of 3-OH-PPA (data not shown). Since the accumulation of 3-OH-PPA could not be quantified by HPLC due to the non availability of authentic standard, the enzyme activity was calculated based on the quantitative determination of *m*-tyrosine disappearance. The enzyme assay further supported the results of resting cells study and confirmed that the first step of *m*-tyrosine degradation occurs by transamination reaction in strain SSC5. The specific activity for the transaminase enzyme was found to be 4.9±0.17 nmol min^−1^ mg of protein^−1^. No transamination activity was observed in the control reactions that lacked either α-KG or cell-free lysates prepared from cells of strain SSC5 grown on *m*-tyrosine or glucose.

### 3-Hydroxyphenylacetate-6-hydroxylase activity

Adding an additional hydroxyl group (-OH) on C-6 of the 3-OH-PhAc ring would result in the formation of HMG [38], [39]. Therefore, identification of HMG intermediate during the resting cell study clearly indicates the involvement of hydroxylation reaction in the conversion of 3-OH-PhAc to HMG. Previous studies have demonstrated that the formation of HMG from 3-OH-PhAc occurs by the action of 3-hydroxyphenylacetate-6-hydroxylase [38], [39]. Enzyme assay using the cell-free lysates prepared from *m*-tyrosine grown cells of strain SSC5 showed hydroxylase activity on 3-OH-PhAc with the formation of HMG as a product. The specific activity of hydroxylase enzyme was found to be 3.20±0.13 nmol min^−1^ mg of protein^−1^. The above experiment provided clear evidence on the involvement of a NADH-dependent hydroxylation reaction in the third step of *m*-tyrosine degradation by strain SSC5.

### Homogentisate 1, 2-dioxygenase activity

To validate the funneling of 3-OH-PhAc into the HMG central pathway (i.e. the fourth step of *m*-tyrosine degradation), an enzyme assay for homogentisate 1, 2-dioxygenase was carried out using the cell-free lysate prepared from the *m*-tyrosine and 3-OH-PhAc grown cells, respectively. The cell-free lysates prepared from 3-OH-PhAc grown cells showed slightly higher 1, 2-dioxygenase activity as compared to the lysates prepared from the cells grown in presence of *m*-tyrosine (Figure 7). The specific enzyme activity was found to be 28.57±0.32 nmol min^−1^ mg of protein^−1^ when grown on 3-OH-PhAc and 26.32±0.15 nmol min^−1^ mg of protein^−1^ when grown on *m*-tyrosine.

The article "Biodegradation of the Allelopathic Chemical m-Tyrosine by Bacillus aquimaris SSC5 Involves the Homogentisate Central Pathway" was retracted in 2014. Reasons: fabricated or falsified data; fabricated or falsified results; concerns about the data.

**Figure 7:** Homogentisate (HMG) 1, 2-dioxygenase activity from the cell-free lysates prepared from *m*-tyrosine-induced cells of strain SSC5. HMG 1, 2-dioxygenase activity was measured by maleylacetoacetate (MA) formation at 330 nm absorbance from cell-free lysates in spectrophotometer. (•), *m*-tyrosine grown cells; (○), 3-OH-PhAc grown cells; (▪), glucose grown cells.

It is known that the homogentisate 1, 2-dioxygenase enzyme transforms HMG to maleylacetoacetate (MA) as a result of ring cleavage of HMG [38], [42]. The cell-free lysates prepared from the cells grown with glucose did not show any dioxygenase activity. Similarly, no dioxygenase activity was observed in the control reactions that lacked cell-free lysates. The above results proved that the homogentisate 1, 2-dioxygenase involved in the homogentisate central pathway, is inducible in nature in the presence of the parent substrate as well as the respective intermediates. Our findings are in close agreement with the results of Mandez et al. [42], who reported 1, 2-dioxygenase activity in the cell-free lysates prepared from 3-OH-PhAc grown cells of *Burkholderia xenovorans* LB400.

## Discussion

Allelopathy is an important mechanism for the competitive advantage of several plants by exudation of various phytotoxic molecules from their roots [1], [53], [54]. The phytotoxic levels of allelochemicals are primarly influenced by process such as their sorption on soil particles and their chemical decomposition. However, soil microbes can also affect the outcome of allelopathic interaction between plants by degrading the released allelochemicals [3], [23], [24], [55]. Kaur et al. [3], have also reported that the outcome of allelopathic interactions of *m*-tyrosine in sterilized soil with a particular species was significantly diminished when non-sterile soil was used. Our microcosm studies showed that the soil microorganisms rapidly degrade *m*-tyrosine in carbon-amended as well as unamended soil (Figure 1). This study showed that soil microbes influence the phytotoxic properties of *m*-tyrosine either by utilizing it as sole carbon, and nitrogen source or transforming it into nontoxic products. Strain SSC5 isolated from the soil microcosms was able to utilize *m*-tyrosine as the sole carbon, nitrogen, and energy source under aerobic conditions. The degradation pathway of *m*-tyrosine in this bacterium has been proposed based on the metabolites identified during the growth and resting cell studies and the enzyme assays (Figure 8). Previous studies have shown that the degradation of L-tyrosine in eukaryotes and prokaryotes occurs by a common peripheral pathway i.e. formation of 4-OH-PPA through the transamination reaction, which funnels into either the HMG or the HPC central pathway [38], [42], [52], [56], [57], [58]. The initial step of *m*-tyrosine degradation occurs with the removal of amino substituent by the action of transaminase activity as determined in crude cell lysates, which is closely similar to the results of Nishino and Spain [36]. They identified 4-hydroxy-3-nitrophenylacetate instead of 4-hydroxy-3-nitrophenylpyruvate from 3-nitrotyrosine by the transamination reaction due to the non-availability of a standard. The GC-MS and ^1^H-NMR analysis of the samples collected from the resting cell study and the transaminase enzyme assay confirmed the formation of 3-OH-PPA as the first metabolic intermediate. Earlier reports have shown that the second step of L-tyrosine degradation is the transformation of 4-OH-PPA into the HMG intermediate with the removal of CO_2_ by the action of 4-hydroxyphenylpyruvate dioxygenase [38], [59]. However, with the identification of the 3-OH-PhAc intermediate in the resting cell study it is presumed that the second degradation step involves the conversion of 3-OH-PPA to 3-OH-PhAc, possibly via a coupled decarboxylation-mooxygenation reaction unlike 4-hydroxyphenylpyruvate dioxygenase which mediates a decarboxylation coupled to a dioxygenation. The decarboxylase enzyme assay from the crude cell lysates could not be carried out due to the non-availability of a 3-OH-PPA standard. During the resting cell study on 3-OH-PhAc, *m*-tyrosine-induced cells transformed 3-OH-PhAc into HMG and this observation was also supported by the NADH-dependent hydroxylase enzyme assay. The results of the hydroxylase activity assay are in close agreement with the results reported earlier [40], [42].

The article "Biodegradation of the Allelopathic Chemical m-Tyrosine by Bacillus aquimaris SSC5 Involves the Homogentisate Central Pathway" was retracted in 2014. Reasons: fabricated or falsified data; fabricated or falsified results; concerns about the data.

**Figure 8:** Proposed metabolic pathway for aerobic degradation of *m*-tyrosine by *Bacillus aquimaris* SSC5. Based on the data from our study, 3-OH-PPA, 3-OH-PhAc, and HMG are identified as the metabolic intermediates during degradation of *m*-tyrosine.

The homogentisate is not the central bacterial catabolic pathway for the degradation of phenylacetic acid and phenylalanine, but it is employed by bacteria for the degradation of hydroxylated phenylacetic acid derivatives and, in rare cases, for phenylalanine [38], [42], [60], [61]. The homogentisate central pathway involves three successive catabolic enzymes i.e. homogentisate 1, 2-dioxygenase, isomerase, and hydrolase, respectively. Homogentisate 1, 2-dioxygenase cleaves the HMG ring and forms MA that is subsequently isomerized by the isomerase enzyme into fumarylacetoacetate (FA) [38]. Further, FA is transformed into fumarate and acetoacetate by the action of a hydrolase [38]. Homogentisate 1, 2-dioxygenase enzyme assays with the cell-free lysates prepared from *m*-tyrosine grown cells showed the conversion of HMG to MA. These data are in close agreement with the results reported earlier [38], [42]. Based on the above studies, it is proposed that the degradation of *m*-tyrosine by strain SSC5 occurs through the HMG central pathway via the formation of 3-OH-PPA and 3-OH-PhAc as major intermediates. The *m*-tyrosine degradation pathway proposed by us is similar to the pathway of L-tyrosine degradation reported earlier in a few bacterial isolates [45], [58], [62], [63].

## Conclusion

This is the first report on metabolism of *m*-tyrosine by *Bacillus aquimaris* SSC5, isolated from soil microcosms. The strain SSC5 utilizes *m*-tyrosine as the sole carbon, nitrogen, and energy source under aerobic conditions. The degradation of *m*-tyrosine occurs with the formation of 3-OH-PPA, 3-OH-PhAc, and HMG as intermediates. The initial step of *m*-tyrosine degradation occurs by the transamination of the amino substituent with the formation of 3-OH-PPA as the first metabolite. Subsequent degradation occurs with the formation of 3-OH-PhAc and HMG as intermediates. Finally, the HMG produced, degrades to MA catalyzed by homogentisate 1, 2-dioxygenase. The present study has significant implications in terms of understanding the environmental fate of *m*-tyrosine and also the masking effect of soil microorganisms over its allelopathic effect. Further studies are needed to establish the regulation and biochemistry of non-proteinogenic amino acid metabolic pathway in *Bacillus aquimaris* SSC5.
